The article "Additional Benefits Conferred by Endoscopic Sclerotherapy to Liver Cirrhosis Patients Receiving Endoscopic Variceal Ligation" was retracted in 2023. Reasons: unreliable results or conclusions; concerns about the data; concerns about the peer review; concerns about the citations.

# Additional Benefits Conferred by Endoscopic Sclerotherapy to Liver Cirrhosis Patients Receiving Endoscopic Variceal Ligation

**DOI:** 10.1155/2021/1294410

**Published:** 2021-10-18

**Authors:** Xuni He, Hanqing Chen, Mingming Zhang, Jiemin Hong, Peina Shi

**Affiliations:** Gastroenterology Department, Ningbo Yinzhou No. 2 Hospital, Zhejiang, China

## Abstract

**Objective:**

Gastroesophageal varices are a direct consequence of portal hypertension in cirrhosis. The management of gastroesophageal varices has evolved over the last decade resulting in reduced mortality and morbidity rates. The study was aimed to analyze the short-term and long-term efficacy of different endoscopic methods in the treatment of gastric varices in cirrhotic patients.

**Methods:**

From January 2016 to December 2019, 135 patients with liver cirrhosis and gastric varices undergoing different endoscopic treatment protocols were retrospectively analyzed. The patients were divided into three groups according to endoscopic variceal ligation, endoscopic sclerotherapy, and a combination of both, respectively. Main outcomes including the overall response rate, hemostasis, short- and long-term rebleeding (3 months before and after treatment), complication, blood pressure, heart rate, portal venous pressure (PVP), portal vein diameter (PVD), portal vein velocity (PVV), portal vein blood flow (PVF) detected by ultrasound, recurrence rate, and mortality were analyzed after treatments.

**Results:**

The overall response rate in the combined group was higher than that in the ligation group and the sclerotherapy group (*P* < 0.05). The incidence rate of complications in the combined group and the ligation group was lower than that in the sclerotherapy group (*P* < 0.05). After treatment, the PVP, PVD, and PVF were reduced in the combined group compared with the ligation group and the sclerotherapy group, while the PVV was not (*P* < 0.05). Lower rates of long-term rebleeding, recurrence, and mortality were noted in the combined group compared to the ligation group and the sclerotherapy group (*P* < 0.05).

**Conclusion:**

Endoscopic variceal ligation combined with endoscopic sclerotherapy is more effective than both alone in treating liver cirrhosis and gastric varices. The combined therapy contributed to reduced short-term and long-term rebleeding rate, decreased long-term recurrence rate, and mortality.

## 1. Introduction

Liver cirrhosis histologically is a diffuse liver injury characterized by fibrosis, with normal structure transformed into abnormal nodules, finally causing pronounced distortion of hepatic vascular architecture [1]. Clinically, liver cirrhosis is considered as a terminal-stage disease, which leads to death in the absence of liver transplantation treatment. The only prevention strategy is to screen esophageal varices, gastric varices, and hepatocellular carcinoma [2]. In the late stage, liver cirrhosis is often characterized by portal hypertension and liver synthesis dysfunction [3]. Portal hypertension in patients with liver cirrhosis leads to various complications, such as esophageal varices, gastric varices, portal hypertensive gastropathy, ascites, and hepatorenal syndrome [4].

The article "Additional Benefits Conferred by Endoscopic Sclerotherapy to Liver Cirrhosis Patients Receiving Endoscopic Variceal Ligation" was retracted in 2023. Reasons: unreliable results or conclusions; concerns about the data; concerns about the peer review; concerns about the citations.

Gastric varices are serious manifestations, which can lead to a large number of gastrointestinal bleeding. Gastric varices often occur in the submucosa of the cardia or gastric fundus, and their location is consistent with the boundary line of portal systemic shunt [5]. The classification of gastric varices commonly used in clinical research was proposed by Sarin and Hashizume. Sarin indicated that the diagnosis was based on the anatomical continuation of esophageal varices and their location in the stomach [6]. However, Hashizume pointed out the classification that was set according to the endoscopic findings of gastric varices, involving form, location, and color [7]. Although the incidence of gastric variceal bleeding is around 10%–36%, which is relatively low compared to esophageal varices, once it occurs, the amount of bleeding is massive which increases the mortality of patients [5].

Some recent advances in drugs and technology have improved the results of gastric varices bleeding, but there is no consensus on the best treatment. In general, endoscopic therapy is the first choice for gastric varices [8]. Endoscopic sclerotherapy has been effective in the treatment of bleeding and eradication in esophageal varices [9]. However, it has been less effective in the treatment of gastric varices, which might due to the high volume of blood flow through gastric varices compared with esophageal varices, with the result of rapid flushing away of the sclerosant in blood. Endoscopic variceal ligation has been commonly used in the treatment of esophageal variceal bleeding [10, 11]. However, few studies referring to the endoscopic variceal ligation or combination of endoscopic sclerotherapy and endoscopic variceal ligation have been found in the treatment of gastric varices. In this study, 135 liver cirrhosis patients with gastric varices were assigned into three groups to analyze the efficacy of endoscopic sclerotherapy, endoscopic variceal ligation, and a combination of both, which might provide supplementary basis for clinical treatment.

## 2. Materials and Methods

### 2.1. Eligible Research Subjects

This study collected and analyzed the clinical data from 135 patients who were admitted into Ningbo Yinzhou No. 2 Hospital from January 2016 to December 2019 for treating liver cirrhosis with gastric varices. According to different endoscopic treatment protocols, endoscopic variceal ligation and endoscopic sclerotherapy alone or combination, 135 patients were divided into the ligation group, sclerotherapy group, and combined group. All patients were examined by liver function tests and transabdominal ultrasound, fulfilling the guidelines for the prevention and management of gastroesophageal varices and variceal hemorrhage in cirrhosis [12]. In addition, age more than 18 years and no less than 3 months of estimated survival time after treatment were also regarded as inclusion criteria. Those patients who met the following criteria were excluded: upper gastrointestinal bleeding caused by nongastric varices, such as esophageal varices, primary liver cancer or other malignancies, noncirrhotic portal hypertension, intolerance to endoscopy or previous failure to endoscopy, allergic to study drugs, and mental or cognitive impairment. The baseline characteristics of included patients are listed in Table 1. The three groups were comparable given that no significant difference was noted on gender, age, the number of gastric varices, Child–Pugh scores, the severity of gastric varices, and duration of liver cirrhosis (*P* > 0.05). This study was approved by the Hospital Ethics Committee. All patients were informed and signed informed consent.

The article "Additional Benefits Conferred by Endoscopic Sclerotherapy to Liver Cirrhosis Patients Receiving Endoscopic Variceal Ligation" was retracted in 2023. Reasons: unreliable results or conclusions; concerns about the data; concerns about the peer review; concerns about the citations.

### 2.2. Treatment Protocols

All patients received general anesthesia before gastroscopy. A gastroscope (LUCERA CV-260, electronic gastroscope GIT-Q260J, Olympus, JPN) was used to explore the position, size, number, severity, and bleeding site of varices. For the patients in the ligation group, a band ligation device was installed after withdrawal of gastroscope and then band ligation was performed with a Saeed six-shooter multiband ligator (MBL-6-F, COOK, USA) after the insertion of gastroscope. From 1-2 cm above the dentate line of the esophagus, the varices were ligated successively by dense ligation from the top to bottom. Each varicose vein was ligated with 3-4 rings, and the distance between adjacent ligation points was about 2-3 cm. Once there was no bleeding, the ligation at the next point was carried out to ensure that each ligation point was not on the same horizontal plane, so as to avoid multiple ligated polypoid varices blocking the food lumen, leading to dysphagia. Do not ligate if the diameter of varicose vein is too large (>1 cm) or the vascular tension is too high. Each patient was ligated with 6–11 rings.

The patients in the sclerotherapy group was injected (injection needle, M00518300, Boston Scientific, USA) with lauromacrogol (National Approval No. H20080445, specification: 10 ml : 100 mg, Shaanxi Tianyu Pharmaceutical Co., Ltd., China) around the bleeding site. In the absence of active bleeding, the injection was performed to varices at 2.5 cm from the upper edge of the Z-line, with 3–5 ml dosage for each site and injection angle within 30°. The total injection dosage was no more than 30 ml. The procedure was finished after irrigation of all sites and confirmation of nonbleeding.

The article "Additional Benefits Conferred by Endoscopic Sclerotherapy to Liver Cirrhosis Patients Receiving Endoscopic Variceal Ligation" was retracted in 2023. Reasons: unreliable results or conclusions; concerns about the data; concerns about the peer review; concerns about the citations.

The patients in the combined group were firstly treated with endoscopic variceal ligation. The specific procedure was the same as the ligation group, and the distance of two ligation sites was kept within 5 cm. Lauromacrogol injection was conducted within the distance. The total injection dosage was not exceeded 10 ml. Irrigation of all sites and confirmation of nonbleeding were done before ending up the therapy.

After endoscopic treatment protocols, the patients in the three groups were forbidden to eat and drink and given additional care, such as hemostasis, acid inhibition, anti-infection, and nutritional support. The patients were given antidrugs to portal hypertension if necessary. During this period, the patient's bleeding and changes of vital signs were closely attended. Feeding was started according to actual situation of patients.

### 2.3. Outcome Measures

Main outcomes including the overall response rate, hemostasis, short- and long-term rebleeding (3 months before and after treatment), complication, blood pressure, heart rate, portal venous pressure (PVP), portal vein diameter (PVD), portal vein velocity (PVV), portal vein blood flow (PVF) detected by ultrasound, recurrence rate, and mortality were analyzed after treatments. Evaluation criteria were as follows: (1) hemostasis referred to the absence of active bleeding, stable vital signs, and no rebleeding within 72 hours after therapy, and hemostasis rate = successful cases/overall cases × 100%; (2) rebleeding referred to the recurrence of hematemesis or black stool caused by gastric varices found by gastroscopy, and rebleeding rate = rebleeding cases/overall cases × 100%; (3) recurrence referred to the presence of varices after elimination, or enlargement of veins that need to be ligated, and recurrence rate = recurrence cases/overall cases × 100%; and (4) treatment response included excellent response, good response, and nonresponse; excellent response meant the changes from block mass or nodositas to cord shape as well as shrinking by more than 50% or disappearance of varices, good response referred to the improvement to a certain extent but the shrinking was no less than 50%, and nonresponse related to no improvement on varices; overall response rate = (excellent response + good response)/overall cases × 100%. All patients were re-examined at 1 month, 3 months, 6 months, and 12 months after therapy, and the re-examination results were recorded. The data within 3 months were defined as the short-term result, and the data after 3 months were considered as the long-term result.

The article "Additional Benefits Conferred by Endoscopic Sclerotherapy to Liver Cirrhosis Patients Receiving Endoscopic Variceal Ligation" was retracted in 2023. Reasons: unreliable results or conclusions; concerns about the data; concerns about the peer review; concerns about the citations.

### 2.4. Statistical Analysis

SPSS20.0 software was used for data processing. The counting data were described by rate/ratio using the chi-square test. The measurement data were expressed as mean ± standard deviation, and the comparison between groups was tested by the *t*-test. *P* < 0.05 indicated that the difference was statistically significant.

## 3. Results

### 3.1. A Better Response after Endoscopic Variceal Ligation and Sclerotherapy

Each patient was followed up 3 months after endoscopic variceal ligation or endoscopic sclerotherapy alone or in combination. The results indicated that the overall response rate in the combined group was higher than that in the ligation group and the sclerotherapy group (*P* < 0.05; Table 2), but no significant difference was observed between the ligation group and the sclerotherapy group (*P* > 0.05).

### 3.2. Rapid Hemostasis and Lower Incidence Rates of Short-Term Rebleeding after Endoscopic Variceal Ligation and Sclerotherapy

As listed in Table 3, there were no significant differences in the incidence rate of complications between the combined group and the ligation group (*P* > 0.05), but they were lower than those in the sclerotherapy group (*P* < 0.05). The hemostasis rate within 72 hours in the combined group was higher than that in the ligation group and sclerotherapy group, and the incidence rate of short-term rebleeding was lower than that in the ligation group and sclerotherapy group. No significant difference was revealed in the hemostasis rate and incidence rate of short-term rebleeding between the ligation group and the sclerotherapy group (*P* > 0.05).

### 3.3. Hemodynamics after Endoscopic Variceal Ligation and Sclerotherapy

It was found that no significant difference was demonstrated in the blood pressure and heart rate among the ligation group, the sclerotherapy group, and the combined group (*P* > 0.05; Table 4). After treatment, the PVP, PVD, and PVF were reduced in the combined group compared with the ligation group and the sclerotherapy group, while the PVV was not (*P* < 0.05). There was no evident difference regarding PVP, PVD, PVV, and PVF between the ligation group and the sclerotherapy group (*P* > 0.05; Table 5).

### 3.4. Lower Incidence Rates of Long-Term Rebleeding, Recurrence Rate, and Mortality after Endoscopic Variceal Ligation and Sclerotherapy

With regard to long-term rebleeding after different endoscopic treatment protocols, it was found that the combined group showed a remarkable lower rate of long-term rebleeding (*P* < 0.05). At the same time, lower recurrence rates and mortality were noted in the combined group compared to the ligation group and the sclerotherapy group (*P* < 0.05; Table 6), but these outcomes revealed no significant difference between the ligation group and the sclerotherapy group (*P* > 0.05).

The article "Additional Benefits Conferred by Endoscopic Sclerotherapy to Liver Cirrhosis Patients Receiving Endoscopic Variceal Ligation" was retracted in 2023. Reasons: unreliable results or conclusions; concerns about the data; concerns about the peer review; concerns about the citations.

## 4. Discussion

Liver cirrhosis is regarded as an advanced chronic liver disease with many complications. In the late stage, it is characterized by portal hypertension [2]. Because of the increased pressure in the portal vein, a variety of complications may occur, including esophageal and gastric varices, ascites, hepatic encephalopathy, and complications secondary to circulatory dysfunction, such as hepatorenal syndrome, portal pulmonary syndrome, and hepatopulmonary syndrome [13, 14]. Varices are preexisting or newly formed portal vein channel expansion, which are common in esophageal and gastric areas at risk of gastrointestinal bleeding [15]. Although the incidence of gastric varices was lower than that of esophageal varices [16] and only 10–30% of variceal bleeding was associated with gastric varices, it was related to higher blood transfusion requirements, uncontrolled bleeding, rebleeding, and death [17, 18]. It was reported that, for the gastric varices patients without bleeding at diagnosis, the cumulative bleeding rates of one-, three-, and five-year follow-up were 4.8%, 19.9%, and 23.2%, respectively [16, 19]. Therefore, it is essential to control bleeding effectively which improves survival rate and reduces mortality.

The condition is dangerous once gastric varices rupture. In recent years, endoscopic therapy has gradually become the primary prophylaxis against bleeding of gastric varices. Endoscopic variceal ligation [20] and endoscopic sclerotherapy [21] have been widely used in variceal bleeding. However, both of them are prone to rebleeding and recurrence after the treatment. In this study, combination of endoscopic variceal ligation and endoscopic sclerotherapy applying to gastric varices in the liver cirrhosis patients was analyzed.

Endoscopic variceal ligation was introduced as a therapeutic option in 1986 [22]. The principle of endoscopic variceal ligation is to inhale the gastric varices into the transparent cap with negative pressure, and then a leather ring is used to ligate the varices in sections to make them ischemic necrosis and form scar tissue, so as to interrupt blood flow [23]. Endoscopic sclerotherapy refers to injecting sclerosant into blood vessel to make varices adhere, resulting in thrombosis and hemostasis [24]. In this study, the data showed that compared to the ligation group and the sclerotherapy group, the combined group showed significant higher overall response rate and hemostasis rate within 72 hours and lower short-term and long-term rebleeding rate, recurrence rate, and mortality. The results of this study were similar to those reported by Li et al. indicating that the combination of ligation and sclerotherapy can improve the therapeutic efficacy and reduce postoperative complications [25].

The article "Additional Benefits Conferred by Endoscopic Sclerotherapy to Liver Cirrhosis Patients Receiving Endoscopic Variceal Ligation" was retracted in 2023. Reasons: unreliable results or conclusions; concerns about the data; concerns about the peer review; concerns about the citations.

The mechanism might be that endoscopic variceal ligation is only associated with thrombosis and occlusion of varices, which has little impact on the pressure in varices, leading to easy falling of the ligation ring used for severe varices. Endoscopic sclerotherapy eliminates varices by chemical methods, which might cause ulcer. At the same time, after sclerosant injection, the collateral circulation of portal vein is blocked, which increases the pressure during left gastric vein shunt, portal vein blood flow, and portal hypertension, with the result of increased bleeding rate and recurrence rate [23, 26]. The combination of the two complements each other to achieve the purpose of rapid hemostasis and blocking collateral circulation, resulting in reduced recurrence and rebleeding.

Endoscopic sclerotherapy is a chemical treatment, which is easy to cause complications such as fever and chest pain. In contrast, endoscopic variceal ligation has fewer complications [27]. The incidence of complications in the present study showed that there was no significant difference between the combined group and the ligation group, but these two groups indicated lower incidence than the sclerotherapy group. The outcomes might be related to the two factors. The one is that, at first, venous route is interrupted and the local blood flow is stopped by endoscopic variceal ligation. It will not cause massive bleeding even if sclerosant is injected into blood vessel. Second, combined treatment refers to injecting sclerosant into the varices along the two ligation sites, which reduces the use of sclerosant, resulting in reduced inflammation and complications. In addition, the results of this study also found that there was no significant difference in blood pressure and heart rate among the three groups before and after therapy, indicating that the three therapies are with high safety.

In summary, the clinical efficacy of combination of endoscopic variceal ligation and sclerotherapy in the treatment of gastric varices is better than these two therapies alone. The combined therapy is associated with rapid hemostasis, reduced recurrence and rebleeding rate, and decreased mortality, which is worthy of promotion in clinical applications. However, the limitations of small sample size and short observation time might lower the reliability of experimental data.

The article "Additional Benefits Conferred by Endoscopic Sclerotherapy to Liver Cirrhosis Patients Receiving Endoscopic Variceal Ligation" was retracted in 2023. Reasons: unreliable results or conclusions; concerns about the data; concerns about the peer review; concerns about the citations.

## Figures and Tables

**Table 1:** Baseline characteristics of the three groups.

Characteristics	Ligation group (*n*)	Sclerotherapy group (*n*)	Combined group (*n*)	*χ* ^2^	*P*
Male/female	26/19	25/20	27/18	0.182	0.913
Age (year)	54.12 ± 8.67	53.69 ± 8.41	54.08 ± 8.36	0.035	0.965
Number of gastric varices (piece)	3.12 ± 0.64	3.14 ± 0.23	3.15 ± 0.37	0.053	0.949
Child–Pugh score	8.21 ± 1.24	8.20 ± 1.17	8.21 ± 1.24	0.003	0.997
Severity of gastric varices (case)				0.184	0.915
F2	24	23	25		
F3	21	22	20		
Cause of liver cirrhosis				0.193	0.956
Hepatitis B	26	25	26		
Alcoholic cirrhosis	19	20	19		
Duration of liver cirrhosis (year)	5.84 ± 1.64	5.82 ± 1.88	5.83 ± 1.76	0.001	0.999

**Table 2:** Comparison of the overall response rate among the three groups.

Group	Excellent response (*n* (%))	Good response (*n* (%))	Nonresponse (*n* (%))	Overall response rate (%)
Ligation group (*n* = 45)	20 (44.44)	16 (35.56)	9 (20.00)	36 (80.00)
Sclerotherapy group (*n* = 45)	19 (42.22)	18 (40.00)	8 (17.78)	37 (82.22)
Combined group (*n* = 45)	28 (62.22)	15 (33.33)	2 (4.44)	43 (95.56)
*χ* ^2^/*P* (ligation vs. sclerotherapy)				0.073/0.788
*χ* ^2^/*P* (ligation vs. combined)				5.075/0.024
*χ* ^2^/*P* (sclerotherapy vs. combined)				4.050/0.044

**Table 3:** The hemostasis rate within 72 hours, incidence rate of complications, and short-term rebleeding rate among three groups after treatment.

Group	Hemostasis rate (*n* (%))	Complications (*n* (%))	Short-term rebleeding (*n* (%))
Ligation group (*n* = 45)	38 (84.44)	5 (11.11)	11 (24.44)
Sclerotherapy group (*n* = 45)	36 (80.00)	13 (28.89)	9 (20.00)
Combined group (*n* = 45)	45 (100.00)	5 (11.11)	4 (8.89)
*χ* ^2^/*P* (ligation vs. sclerotherapy)	0.304/0.581	4.444/0.035	0.257/0.612
*χ* ^2^/*P* (ligation vs. combined)	7.590/0.006	0.000/1.000	3.920/0.048
*χ* ^2^/*P* (sclerotherapy vs. combined)	10.000/0.002	4.444/0.035	2.248/0.134

**Table 4:** The blood pressure and heart rate among three groups before and after treatment.

Group	Before treatment			After treatment		
	Systolic pressure (mmHg)	Diastolic pressure (mmHg)	Heart rate (times/min)	Systolic pressure (mmHg)	Diastolic pressure (mmHg)	Heart rate (times/min)
Ligation group (*n* = 45)	121.31 ± 10.14	82.04 ± 10.11	79.21 ± 10.32	120.42 ± 10.21	80.12 ± 10.27	80.11 ± 10.18
Sclerotherapy group (*n* = 45)	120.24 ± 10.37	81.21 ± 10.14	78.24 ± 10.54	119.21 ± 10.24	80.17 ± 10.19	79.21 ± 10.23
Combined group (*n* = 45)	121.58 ± 10.42	80.34 ± 10.26	78.23 ± 10.21	120.37 ± 10.36	80.28 ± 10.22	79.65 ± 10.47
*t*/*P* (ligation vs. sclerotherapy)	0.495/0.622	0.389/0.698	0.441/0.660	0.561/0.576	0.023/0.982	0.418/0.677
*t*/*P* (ligation vs. combined)	0.125/0.901	0.792/0.431	0.453/0.652	0.023/0.982	0.074/0.941	0.211/0.833
*t*/*P* (sclerotherapy vs. combined)	0.611/0.543	0.405/0.687	0.005/0.996	0.534/0.595	0.051/0.959	0.202/0.841

The article "Additional Benefits Conferred by Endoscopic Sclerotherapy to Liver Cirrhosis Patients Receiving Endoscopic Variceal Ligation" was retracted in 2023. Reasons: unreliable results or conclusions; concerns about the data; concerns about the peer review; concerns about the citations.

**Table 5:** The PVP, PVD, PVV, and PVF among the ligation group, the sclerotherapy group, and the combined group before and after treatment.

	PVP	PVD	PVV	PVF
Ligation group (*n* = 45)	25.37 ± 2.03	13.84 ± 0.47	20.25 ± 4.32	741.82 ± 158.45
Sclerotherapy group (*n* = 45)	24.85 ± 1.92	14.14 ± 0.51	21.03 ± 4.72	752.36 ± 163.15
Combined group (*n* = 45)	21.45 ± 1.67	11.43 ± 0.35	19.93 ± 4.22	539.59 ± 128.41
*t*/*P* (ligation vs. sclerotherapy)	1.248/0.215	2.902/0.005	0.416/0.818	0.311/0.757
*t*/*P* (ligation vs. combined)	10.000/<0.001	27.590/<0.001	0.723/0.356	6.652/<0.001
*t*/*P* (sclerotherapy vs. combined)	8.963/<0.001	29.390/<0.001	1.165/0.247	6.875/<0.001

**Table 6:** The long-term rebleeding rate, recurrence rate, and mortality among three groups after treatment.

Group	Long-term rebleeding (*n* (%))	Recurrence rate (*n* (%))	Mortality (*n* (%))
Ligation group (*n* = 45)	18 (40.00)	13 (28.89)	8 (17.78)
Sclerotherapy group (*n* = 45)	19 (42.22)	14 (31.11)	7 (15.56)
Combined group (*n* = 45)	6 (13.33)	5 (11.11)	1 (2.22)
*χ* ^2^/*P* (ligation vs. sclerotherapy)	0.046/0.830	0.053/0.818	0.080/0.777
*χ* ^2^/*P* (ligation vs. combined)	8.182/0.004	4.444/0.035	6.049/0.014
*χ* ^2^/*P* (sclerotherapy vs. combined)	9.360/0.002	5.404/0.020	4.939/0.026

## Data Availability

The data used to support the findings of this study are included within the article.
